RETRACTED

# Comparison of Clinical Efficacy of Sodium Nitroprusside and Urapidil in the Treatment of Acute Hypertensive Cerebral Hemorrhage

**DOI:** 10.1155/2022/2209070

**Published:** 2022-03-28

**Authors:** Rui Yang, Zhenzhen Wang, Yanxun Jia, Hao Li, Yating Mou

**Affiliations:** ^1^Department of Neurology, Gucheng Hospital, Hengshui 253800, China; ^2^Department of Neurosurgery, Gucheng Hospital, Hengshui 253800, China

## Abstract

This paper mainly studies the clinical efficacy of sodium nitroprusside and urapidil in the treatment of acute hypertensive intracerebral hemorrhage and analyzes the brain CT image detection based on a deep learning algorithm. A total of 132 cases of acute hypertension admitted to XXX hospital from XX 2019 to XX 2020 were retrospectively analyzed. The diseases of all patients were clinically confirmed, and patients were divided into groups according to the differences in treatment methods. Urapidil was used for group 1; sodium nitroprusside was used for group 2; and urapidil combined with sodium nitroprusside was used for group 3. A convolutional neural network in deep learning is used to construct intelligent processing to classify brain CT images of patients. The network performance of AlexNet, GoogLeNet, and CNN3 is predicted. The results show that GoogLeNet has the highest prediction accuracy of 0.83, followed by AlexNet with 0.80 and CNN3 with 0.74. The results of the performance parameter curve show that the GoogLeNet has the highest performance parameter of 0.89, followed by AlexNet and CNN3 network. The performance parameter curve of machine learning is above 0.80. After five weeks of drug treatment, the hematoma volume was (3.8 ± 2.6) mL in group1, (7.6 ± 2.8) mL in group 2, and (2.8 ± 1.5) mL in group 3. After 5 days of treatment, the patients' heart rate changed compared with before treatment. Compared with group 2, there were significant differences between groups 1 and 3 (*P* < 0.01), indicating that the therapeutic effect of the combination group was significantly better than that of the other groups alone. In summary, the combination of sodium nitroprusside and urapidil has a significantly better effect than that of urapidil alone. A convolutional neural network based on deep learning improves the recognition accuracy of medical images.

## 1. Introduction

Hypertensive cerebral hemorrhage (HICH) is a common cerebrovascular disease with high incidence, mortality, and disability, which belongs to the category of “hemorrhage and stroke disease” in traditional Chinese medicine. Stroke disease is proposed from the theory of sputum therapy and is described in Danxi·Xinfa Stroke: “Stroke is mainly characterized by blood deficiency and phlegm. Treatment of phlegm is the priority, and blood cultivation is the second priority” [1]. HICH treatment in the acute stage is quite important, which has a direct impact on patients' quality of life [2]. With the continuous improvement of living standards, the incidence of this disease is increasing. At present, hypertensive intracerebral hemorrhage is one of the three major human death diseases, which brings serious damage to human physical and mental health. According to relevant literature reports, the incidence of a cerebral hemorrhage in the population is 100,000 people/year. In the incidence of foreign countries, cerebral hemorrhage accounts for about 15% of all strokes, and all hospitalized stroke patients account for 10% to 30%. In China, the proportion of patients is 18.8%–47% [3, 4]. HICH acute disease changes rapidly, and the fatality rate is high, especially in the first 2 days of onset [5]. HICH generally occurs in males, aged between 50 and 70 years old, and tends to occur more frequently in winter and spring. Hypertensive diseases will lead to pathological changes in the arterioles at the base of the brain, with prominent manifestations such as hyaloid or fibrous changes and focal hemorrhage, ischemia, and necrosis on the arterioles wall, which weakens the strength of the vascular wall, leads to localized dilation, and may lead to the formation of tiny aneurysms [6, 7]. The onset of HICH is rapid during agitation and activity, and the disease will reach its peak in a few minutes [8, 9]. Patients may experience headaches, nausea, vomiting, agitation, drowsiness, or coma, sometimes with breathing problems, slow pulse, elevated blood pressure, and other symptoms. Aggressive and rational treatment can save lives, reduce neurological disability, and recurrence rate. The main treatment methods include medical treatment, surgical treatment, rehabilitation treatment, and dietary restriction [10, 11].

RETRACTED

CT detection can timely and accurately display the bleeding site, bleeding volume, edema volume around the hematoma, hematoma morphology, and whether the middle line of the brain moves and then determine the secondary bleeding. Minimally invasive blood clearance can also be performed for patients under CT localization [12–14]. Intelligent machine learning for data recognition and analysis is simpler. The traditional classification processor is based on manual, which is not only time-consuming but also has the characteristics of large error and relatively low recognition accuracy, so it can not display the image quality well [15]. If not timely treatment, it is likely to develop into hemiplegia, dementia, and other serious situations, not only affecting patients' quality of life but also bringing a huge burden to patients and their families [16, 17]. Medical technology is also developing rapidly. Although it saves the lives of many patients with brain diseases, many patients will have multiple sequelae after treatment, which seriously affects the prognosis of patients [18]. Deep learning is a new field in machine learning research. An artificial neural network is a kind of deep learning model structure containing multilayer perceptron, and automatic operating procedures are more convenient in magnetic resonance imaging [19, 20]. Oh et al. [21] found that using a computer learning algorithm, combined with CT radiological characteristics and clinical information training model, it can effectively predict the femoral fracture, which has obvious advantages in preventing disease complications. Kim et al. [22] effectively constructed a model to predict the complications of spinal deformity surgery through a computer learning algorithm. The calculation program was improved by American surgeons. The constructed ANN and logistic regression can predict each complication and can also effectively predict the self-management of patients with postoperative complications [23, 24]. In the deep learning model, the convolution neural network is used to segment and classify the human brain CT images, and the intelligent processor in the network is used to extract the image features. After the training data and test data are processed by the convolution neural network, the mapping relationship between the input and the label is obtained, indicating that the parameter model has been trained, and the image is reconstructed.

The proportion of HICH in acute cerebrovascular diseases is 30%, which poses a certain threat to the life safety of patients. However, whether patients with acute hypertensive cerebral hemorrhage should be given active antihypertensive treatment has not been determined. In previous treatments, symptomatic support, anticerebral edema, and blood pressure were selected for control, and the therapeutic effect was not ideal. Sodium nitroprusside can improve myocardial blood supply, reduce blood pressure, and expand blood vessels. Urapidil is a highly selective *α*1-adrenoceptor blocker, which has a good antihypertensive effect on peripheral and central. Therefore, this study applies neural networks to image processing networks. Taking patients with acute hypertensive cerebral hemorrhage as the research object, deep learning convolutional neural network is introduced into CT images to classify CT images intelligently. Then, the effect of sodium nitroprusside and urapidil in the treatment of hypertension in the acute stage of a cerebral hemorrhage was analyzed to provide a theoretical basis for the clinical diagnosis and treatment of HICH, to provide help for clinical diagnosis and treatment.

RETRACTED

## 2. Materials and Methods

### 2.1. Research Objects

A total of 132 cases of acute hypertension admitted to XXX hospital from XX in 2019 to XX in 2020 were selected as the research objects. All patients had clinically proven diseases and were divided into groups based on differences in treatment methods, group 1 (*n* = 44) and group 2 (*n* = 4 4).

Group 2 (33 males and 11 females, from 52 to 70 years old, with an average of (63.24 ± 3.05 years). Group 1 (36 males and 8 females, from 50 to 75 years old, with an average of 65.56 ± 2.74 years. Group 3 (n = 44) (30 males and 14 females. The average age was (59.24 ± 2.36 years) from 55 to 71 years old. There was no statistically significant difference in the general data of patients in the three groups.

Group 1 was treated with urapidil (Shandong Luoxin Pharmaceutical Co. Ltd., H11020907); group 2 was treated with sodium nitroprusside (China Resources Double-Crane Pharmaceutical Co. Ltd., H11020907); and Group 3 was treated with urapidil combined with sodium nitroprusside. The drugs were mixed with 50 mL normal saline at a dose of 200 mg. During the treatment, vital signs such as heart rhythm, respiration, and blood pressure were detected, and then the treatment effect of each group was evaluated and analyzed. The test has been approved by the ethics committee of XXX hospital. All patients and their families understood and signed the informed consent form.

Inclusion criteria are as follows:(1) the patients met the clinical diagnostic criteria of cerebrovascular disease in China and were the first to develop the disease; (2) the patients were confirmed by cranial examination; (3) they had good comprehension and communication skills; and (4) the neuromotor function score of all patients was evaluated by the National Institute of Health Stroke Scale (NIHSS).

Exclusion criteria are as follows:(1) those with a history of mental disorders and those who did not cooperate; (2) patients complicated with other neurological diseases such as Alzheimer's disease and Parkinson's disease; (3) patients with severe cardiac and renal complications that may cause malignant hypertension and increased blood pressure caused by urinary retention, restlessness, and other factors, with systolic blood pressure >200 and diastolic blood pressure >110; and (4) onset time <3.

### 2.2. Index Evaluation

The patients were scored with the NIHSS at the first week after admission and the fifth week after treatment, and then the patients' head CT examination was performed to compare the hematoma volume at the first week and after the fifth week of treatment.

RETRACTED

### 2.3. CT Image Preprocessing

CT image is a series of continuous slices obtained by computer transverse scanning. These slices are combined to form a three-dimensional CT image. CT image is different from natural image. Doctors often judge diseases according to organ texture features, shape features, and spatial relationship in CT image. CT image preprocessing generally includes two methods, one is a morphological method, and the other is to use the existing algorithm for contour extraction. The CT image processing flow of morphology is shown in Figure 1. The threshold is manually set for binarization; then the boundary is cleaned to obtain the maximum connected area; then the double trilinear difference is unified; and finally, the unified standard data is obtained.

### 2.4. CT Scanning Process

Multislice spiral CT examination method includes the following: (1) hip joint scanning. (2) CT setting. The Optima CT600 spiral machine produced by GE company was used to scan the skull image of the patients, and the patients needed respiratory training before scanning. During the examination, the supine position was taken for CT scan, and the whole lung examination was performed when the patient was deeply breathing and breath holding. Setting scan parameters are as follows: 0.875 pitch, 38 × 38 cm field of vision, 512 × 512 matrix, 1,500 window width, −650 U window position, 0.5 cm layer thickness, and 0.5 cm layer spacing. The CT standard reconstruction algorithm is used to reconstruct the CT image, and the thickness of the layer is 0.625 mm, and the spacing is 0.625 mm. The reconstructed CT images were uploaded to the workstation, and the skull indexes were measured by Thoracic VCAR Airway Analysis software. The computer uses a deep learning algorithm to reconstruct the image and retain the image of the patient's lesion. The diagnosis results of the lesion before and after the algorithm are analyzed and compared. The CT images of cerebral hemorrhage were read by three physicians with rich imaging experience in the department of radiology, and the lesions in different parts of each joint were recorded.

### 2.5. Deep Learning Network

A deep learning network includes unsupervised learning and supervised learning. The supervised learning networks include convolutional neural network, cyclic neural network, and recursive neural network. Unsupervised learning includes deep belief network, self-encoder, and generation of confrontation network. Deep learning network has gradually evolved from target detection and classification, and data compression to image segmentation has been widely used in medical images, which has significant effects in image quality assessment and image modal transformation.  Figure 2 presents a basic structure of the convolutional neural network.

RETRACTED

### 2.6. Transfer Learning Network

AlexNet introduces a convolutional neural network into the ILSVRC competition, and the error rate is 17%. The introduction of the modified linear unit activation function in the AlexNet model can effectively shorten the learning cycle. The AlexNet model has 650,000 neurons and 60 million parameters. The structure consists of a softmax layer, three fully connected layers, and five convolution layers. Experimental results show that the training of deep convolutional neural networks with modified linear unit activation functions is several times faster than the same network with tanh units. Network training in two graphics processors can achieve better processing results. AlexNet uses local response normalization function and overlapping pooling to synthesize the output of adjacent neurons in the same kernel mapping.  Figure 3 displays the AlexNet structure of the deep learning network.

### 2.7. Inception Structure of Deep Learning Network GoogLeNet

GoogLeNet is a 27-layer deep learning network with about 500,000 parameters. Compared with the deep 22-layer AlexNet, the optimized parameters are one-twelfth of the AlexNet. Various technical details of convolutional neural networks have been widely studied and improved, including some loss functions, activation functions, and structural units. These networks have been gradually deepened and priced and have been widely used in many fields. GoogLeNet learns from the 1 × 1 convolution method to increase the network depth in technology and draws on the filter for multiscale analysis method in technology. The multilevel analysis method is used to improve the accuracy of network recognition by integrating the feature information of different depths. GoogLeNet is deeper and wider than the AlexNet, but the optimized parameters are less.  Figure 4 shows the inception structure of the deep learning network GooLeNet.

### 2.8. Construction of Convolutional Neural Network Model

The structure of the convolutional neural network includes input layer, convolution layer, downsampling layer, full connection layer, and output layer. The convolution layer includes multiple calculation layers, and each calculation layer contains multiple feature maps. Each feature map represents a specific plane, and the neurons in the same plane have the same weight. The specific convolution equation is as follows:

(1) $$\begin{array}{c} X_{j}^{k}=g\left(\sum_{i\in N_{j}}X_{i}^{k-1}*l_{ij}^{k}+a_{i}^{k}\right), \end{array}$$

where *N*_*j*_ represents the local sensory area of neurons *j*, *X*_*i*_^*k*−1^ represents the output value of neurons *i* in the *k* − 1 layer, *l*_*ij*_^*k*^ represents the *j* weight of neurons *i*, and *a*_*i*_^*k*^ represents the offset number *i* at the *k* layer. The downsampling layer is the feature extraction layer. Assuming that there are *m* feature images, the number of images does not change after the downsampling layer processing, but the size is significantly smaller. The specific calculation equation is as follows:

(2) $$\begin{array}{c} X_{j}^{k}=g\left(\delta^{k}dec\left(z_{i}^{k-1}\right)+a^{k}\right), \end{array}$$

where *dec*() represents the down-sampling, *δ*^*k*^ represents the adjustment parameter, as a constant, and *a*^*k*^ represents the adjustment bias. The full connection layer is closely connected with the upper layer. When the upper layer outputs the results, the full connection layer is calculated by the sigmoid function, and the specific form is as follows:

(3) $$\begin{array}{c} X_{j}^{k}=g\left(\sum_{i\in N_{j}}v_{ji}*X_{i}^{k-1}+a^{k}\right), \end{array}$$

where the weight between the *i* input and the *j* output of the *k* − 1 layer is represented as *v*_*ji*_, and the training bias is represented as *a*^*k*^. Input layer samples determine the type of output layer samples, and the maximum probability of each input layer sample corresponds to the final type of output samples. The random gradient descent method is used to train the algorithm in this study. The basic equation is as follows:

(4) $$\begin{array}{c} \lambda_{j}≔\lambda_{j}-\phi \frac{\partial }{\partial \lambda_{j}}J\left(\lambda \right), \end{array}$$

where *ϕ* represents the learning efficiency, and the step size of gradient descent can be adjusted. If the *ϕ* value is too small, it will lead to the convergence speed of the algorithm being too slow, and if the value is too large, the algorithm cannot converge normally. The value of the algorithm *ϕ* in this study is 0.2. The Gaussian mixture model is used for optimization. Assuming that random variables *X* obey Gaussian distribution *M*(*η*, *σ*^2^), the probability density function of the Gaussian function is expressed as follows:

(5) $$\begin{array}{c} g\left(x\right)=\frac{1}{\sqrt{2\pi }\sigma }\exp\left(-\frac{{\left(x-\eta \right)}^{2}}{2\sigma^{2}}\right), \end{array}$$

where *η* represents a mathematical expectation and *σ*^2^ represents a variance. Probability density function expression of the Gaussian mixture model is as follows:

(6) $$\begin{array}{c} Q\left(x_{i}|\psi \right)=\sum_{l=1}^{L}\pi_{l}Q_{l}\left(x_{i}|\phi_{l}\right), \end{array}$$

where the coefficient *π*_*l*_ representing the Gaussian mixture density function is the weight value of the *l* Gaussian distribution, Ψ represents the parameter vector in the mixed model, *ϕ*_*l*_ represents the Gaussian distribution parameter, and *Q*_*l*_ represents the probability density function of the *l* Gaussian mixture distribution. According to the maximum density function, the size of parameter values can be estimated, generally using the following estimation equation.

(7) $$\begin{array}{c} Q\left(X|\psi \right)=\prod_{i=1}^{M}Q\left(x_{i}|\psi \right)=K\left(\psi |X\right),\\ \psi =\arg\max L\left(\psi |X\right). \end{array}$$

In general, the partial derivative of some variables is used to obtain the maximum value of the function, and the parameters are modified and iterated to converge to the maximum error range.

(8) $$\begin{array}{c} \Delta a=\frac{a_{1}-a}{W},\\ \Delta \text{b}=\frac{b_{1}-\text{b}}{h},\\ \Delta \text{w}=\log\frac{w_{1}}{W},\\ \Delta h=\frac{h_{1}}{h}. \end{array}$$

Feature extraction plays an important role in image information classification.

RETRACTED

### 2.9. Model Training Test

The preprocessing program environment in this article is Ubuntu16.04, and the programming language is Python. Image preprocessing requirement medical image toolkits include SimpleITK, pydicom, and nibabel. SimpleITK reads the CT image of mhd format; nibable is used to read the CT image of nii format; pydicom reads the CT image of dicom format; and ITKSNAK software is used to display the processed image. Then, the contrast is adjusted according to different characteristics of data, and the adjusted parameters are used for batch processing of data.

Two images are processed in the central processor, and four GPUs are selected for training, effective batch 8. The hardware platform parameters of the model are dual 4-core Intel(R) Xeon (R) E5-2623 v4 @ 2.60 GHz processor and 128 GB 4*∗*32 GB 2400 MHz DDR4 ECC Reg memory. Operating environment is as follows: 64-bit Ubuntu16.04.7 operating system and Pytorch_0.4.0 program environment. The AlexNet and GoogLeNet models can be downloaded from Caffe Model Zoo. Based on the downloaded training model, 103 nodes in the final softmax output layer are replaced by 2 nodes for the classification of CT images, and then training, verification, and testing are carried out according to different data sets. The trained features of the convolutional neural network model are input into SVM, and the extracted features include orientation gradient histogram, gradient divergence histogram, gray level co-occurrence matrix, and so on. The basic learning rate of the model is set to 0.001; the momentum is 0.9; the attenuation parameter is 0.0005; and other parameters remain unchanged.

RETRACTED

### 2.10. Statistical Methods

In this study, SPSS21.0 software is used for the statistical analysis of the data. The measurement data in line with normal distribution are expressed by mean ± standard deviation ($\bar{x}$ ± *s*), and the nonconforming counting data are expressed by frequency and frequency rate (%). With *α* = 0.05 as the test level of comparison between groups, when *P* < 0.05, it is considered that the difference is statistically significant.

## 3. Efficacy Data Statistics

### 3.1. Network Performance and Accuracy Prediction

The accuracy of the algorithm is predicted, as shown in Figure 5. GoogLeNet has the highest prediction accuracy of 0.83, followed by AlexNet, with a prediction accuracy of 0.80. CNN3's network prediction accuracy is 0.74, and CNN2's network prediction accuracy is 0.73. The prediction accuracy of deep learning convolutional neural network is significantly higher than that of a shallow convolutional neural network. The classification accuracy of the deep convolution neural network with transfer depth learning is lower than 0.85, and the higher judgment accuracy provides additional auxiliary functions for doctors' decision-making in the clinic.

Figure 6 shows the performance parameter curve of the algorithm. The highest performance parameter of the GoogLeNet is 0.89, followed by the AlexNet and the CNN3. The performance parameter curve of machine learning is above 0.80.

### 3.2. Network Characteristic Curve

The ROC curves of the three auxiliary diagnostic models are shown in Figure 7. In Figure 7, the blue is CNN3; the orange is AlexNet; and the gray is GoogLeNet. It is obvious from Figure 7 that the performance of GoogLeNet is better than the other two networks.

### 3.3. Images of Different Networks

Figure 8 shows the comparison of imaging images of different networks. Figure 8(a) is CT images of the brain in GoogLeNet. Figure 8(b) is CT images of patients with intracerebral hemorrhage in the AlexNet. Figure 8(c) is CT images of patients with intracerebral hemorrhage in the CNN3.

### 3.4. Images

Figures 9(a) and 9(b) are the CT images of cerebral hemorrhage in a 62-year-old male patient, which are caused by rupture of the lenticulostriate artery, especially its lateral branch. The main manifestations are sudden contralateral hemiplegia, hemianesthesia defect, isotropic blindness, and aphasia in the main and lateral hemispheres. A large amount of bleeding can be a conscious disturbance, and a small amount of bleeding only shows pure exercise, without headache vomiting. The number 1 shows hemorrhage in the left capsule, and the number 2 shows calcification in the globus pallidus in Figure 9.

RETRACTED

Figure 10 shows the brain CT manifestations of a 52-year-old male. The figure showed that the symptoms are serious, and the clinical manifestations are diverse and complex, which could lead to multiple clinical symptoms and signs of hemorrhage of the nucleus and thalamus.

Figure 11 shows the brain CT manifestations of a 68-year-old male. A large number of brain hemorrhages involving bilateral caps and bases are often broken into the fourth ventricle, leading to coma, bilateral needle-like pupil, vomiting coffee-like gastric content, central high fever, and central respiratory disorders. Mild cerebral hemorrhage manifested as incomplete paralysis of unilateral or bilateral oculomotor nerve, paralysis of the oculomotor nerve on lesion side, and paralysis of lateral nerve, sublingual nerve, and upper and lower limb motor nerve.

### 3.5. Hematoma Volume in Three Groups

The hematoma volumes of the two groups were compared. The results are shown in Table 1. At the time of treatment, the hematoma volumes of groups 1, 2, and 3 were (32.51 ± 8.3) mL, (33.02 ± 9.2) mL, and (34.52 ± 7.4) mL, respectively. After one week of drug treatment, the hematoma volumes of groups 1, 2, and 3 were (18.6 ± 2.6) mL, (22.8 ± 3.1) mL, and (16.92 ± 3.2) mL, respectively. After five weeks of drug treatment, the hematoma volumes of groups 1, 2, and 3 were (3.8 ± 2.6) mL, (7.6 ± 2.8) mL, and (2.8 ± 1.5) mL, respectively.

### 3.6. Comparison of Heart Rate Changes of the Three Groups before and after Treatment

The heart rate changes of the three groups before and after treatment were analyzed. The results are shown in Figure 12. The heart rates of the three groups after 5 days of treatment were changed compared with those before treatment. Compared with group 2, there was a significant difference between groups 1 and 3 (*p* < 0.01), indicating that the treatment effect of the combined drug group was significantly better than that of other single drug groups.

The heart rate of the three groups changed after 30 days of treatment compared with before treatment. After 30 days of treatment, the difference between groups 2 and 3 was significant (*p* < 0.01), and the difference between group 1 and before treatment was significant.  Figure 13 is a comparison of heart rate changes among the three groups before and after treatment.

## 4. Discussion

HICH is an acute cerebrovascular disease with high morbidity and a high disability rate. Many studies have shown that hematoma enlargement in hypertensive intracerebral hemorrhage within 24 hours is closely related to the maximum systolic blood pressure and average systolic blood pressure but has little relationship with diastolic blood pressure and blood pressure variability. Some researchers believed that hematoma enlargement occurred in 25.4% of patients with cerebral hemorrhage, 41.3% occurred in 2–3 days after the onset, and 14% occurred in 3–4 days after the onset. The aggravation probability of neurological deficit symptoms in patients with hematoma enlargement increased 4 times. Effective and reasonable control of brain hemorrhage is very important for the treatment of acute hypertension. Sodium nitroprusside can reduce blood pressure to expand blood vessels, but there will be accelerated blood reflex heart rate. It is necessary to monitor the blood pressure of patients in real time and control the drip rate according to the actual situation. Sodium nitroprusside can effectively improve the left ventricular function of patients and significantly increase cardiac output. Urapidil can change the sympathetic nerve excitation and regulate the activity of the central nervous system. Exciting the central 5-hydroxytryptamine IA receptor can reduce blood pressure, expand blood vessels, effectively relieve sympathetic pressure, hinder the prominent posterior membrane *α*1 receptor, and ultimately increase cardiac output.

RETRACTED

CNN model belongs to the feedforward neural network and is a multilayer perceptron model constructed to identify two-dimensional and above images. The image information of different modes can give feedback to patients from different levels, different angles, and different modes, which is more conducive to the diagnosis of diseases. The increase of feature dimension directly affects the parameter optimization of classifier and has become a key factor in AI-aided diagnosis. In this study, the first dimension of the softmax layer of AlexNet and GoogLeNet is 4096, and CNN2 and CNN3 are 400 dimensions. Higher feature dimensions are more conducive to building complex mapping functions.

## 5. Conclusion

In order to investigate the clinical efficacy of sodium nitroprusside and urapidil in patients with acute hypertensive cerebral hemorrhage, the brain CT image detection based on a deep learning algorithm was analyzed. Deep learning convolutional neural network can classify CT imaging well. A convolutional neural network can be used to quickly collect data. In network based on deep learning, the processor intelligently extracts the features of lesions. It has the highest prediction accuracy of 0.83 for GoogLeNet of cerebral infarction, followed by AlexNet, and the prediction accuracy is 0.80. The network prediction accuracy of CNN3 is 0.74. The combination effect of sodium nitroprusside and urapidil is significantly better than that of monotherapy. The deep learning convolution network has been constantly updated. In addition to the AlexNet and GoogLeNet mentioned in this study, the deep convolution neural model also has a generative confrontation network, sparse self-coding network, residual network, and so on. In the future, we can have a deeper understanding of the deep learning convolution network in these aspects. Machine learning needs large-scale data model training. The data used in this study are relatively small, and targeted cooperation of multiple research centers can be carried out to obtain large sample medical image data, which can make the deep learning model closer to clinical practice and achieve higher accuracy.

RETRACTED

## Figures and Tables

**Figure 1:** CT image preprocessing process.

**Figure 2:** The basic structure of the convolutional neural network.

**Figure 3:** AlexNet structure of deep learning network.

**Figure 4:** Inception structure of deep learning network GooLeNet.

**Figure 5:** Predictive performance of the diagnostic system.

**Figure 6:** CT images of thalamic hemorrhage.

**Figure 7:** Operating characteristic ROC curve.

**Figure 8:** Comparison of different network CT images.

**Figure 9:** CT image of thalamic hemorrhage.

**Figure 10:** CT image of mixed hemorrhage.

**Figure 11:** CT images of brainstem hemorrhage.

**Figure 12:** Comparison of heart rate changes among the three groups before and after treatment (^*∗*^represents statistically significant difference compared with group 1, *p* < 0.01).

**Figure 13:** Comparison of heart rate changes among the three groups before and after treatment (^*∗*^ represents a statistically significant difference compared with group 1 of sodium nitroprusside, *p* < 0.05, and # represents a statistically significant difference compared with before treatment, *p* < 0.05).

**Table 1:** Hematoma volume after different treatments.

Group	Treatment	First week	Fifth week
Group 1	32.51 ± 8.3	18.6 ± 2.6	3.8 ± 3.6
Group 2	33.02 ± 9.2	22.8 ± 3.1	7.6 ± 2.8
Group 3	34.52 ± 7.4	16.92 ± 3.2	2.8 ± 1.5
*F*	0.128	5.634	3.879
*p*	＞0.05	＜0.001	＜0.001

## Data Availability

The simulation experiment data used to support the findings of this study are available from the corresponding author upon request.
